# Chicoric Acid Ameliorates Nonalcoholic Fatty Liver Disease via the AMPK/Nrf2/NF*κ*B Signaling Pathway and Restores Gut Microbiota in High-Fat-Diet-Fed Mice

**DOI:** 10.1155/2020/9734560

**Published:** 2020-11-03

**Authors:** Xiaoqin Ding, Tunyu Jian, Jiawei Li, Han Lv, Bei Tong, Jing Li, Xiuhua Meng, Bingru Ren, Jian Chen

**Affiliations:** ^1^Institute of Botany, Jiangsu Province and Chinese Academy of Sciences, Nanjing 210014, China; ^2^Department of Food Science and Technology, College of Light Industry and Food Engineering, Nanjing Forestry University, Nanjing 210037, China

## Abstract

This study examines the effects of chicoric acid (CA) on nonalcoholic fatty liver disease (NAFLD) in high-fat-diet- (HFD-) fed C57BL/6 mice. CA treatment decreased body weight and white adipose weight, mitigated hyperglycemia and dyslipidemia, and reduced hepatic steatosis in HFD-fed mice. Moreover, CA treatment reversed HFD-induced oxidative stress and inflammation both systemically and locally in the liver, evidenced by the decreased serum malondialdehyde (MDA) abundance, increased serum superoxide dismutase (SOD) activity, lowered *in situ* reactive oxygen species (ROS) in the liver, decreased serum and hepatic inflammatory cytokine levels, and reduced hepatic inflammatory cell infiltration in HFD-fed mice. In addition, CA significantly reduced lipid accumulation and oxidative stress in palmitic acid- (PA-) treated HepG2 cells. In particular, we identified AMPK as an activator of Nrf2 and an inactivator of NF*κ*B. CA upregulated AMPK phosphorylation, the nuclear protein level of Nrf2, and downregulated NF*κ*B protein level both in HFD mice and PA-treated HepG2 cells. Notably, AMPK inhibitor compound C blocked the regulation of Nrf2 and NF*κ*B, as well as ROS overproduction mediated by CA in PA-treated HepG2 cells, while AMPK activator AICAR mimicked the effects of CA. Similarly, Nrf2 inhibitor ML385 partly blocked the regulation of antioxidative genes and ROS overproduction by CA in PA-treated HepG2 cells. Interestingly, high-throughput pyrosequencing of 16S rRNA suggested that CA could increase *Firmicutes*-to-*Bacteroidetes* ratio and modify gut microbial composition towards a healthier microbial profile. In summary, CA plays a preventative role in the amelioration of oxidative stress and inflammation via the AMPK/Nrf2/NF*κ*B signaling pathway and shapes gut microbiota in HFD-induced NAFLD.

## 1. Introduction

Nonalcoholic fatty liver disease (NAFLD), characterized by hepatic fat accumulation in patients without consumption of excessive alcohol, is the manifestation of metabolic syndrome in the liver. NAFLD ranges from simple hepatic steatosis to steatohepatitis (NASH), fibrosis, and cirrhosis [1]. The prevalence of NAFLD is increasing rapidly worldwide, which has become the major cause of chronic liver disease consistent with the increasing incidence of obesity [2]. The underlying mechanism in the development of NAFLD is complicated. The increase of free fatty acid (FFA) levels could cause fat accumulation, along with consequent oxidative stress and insulin resistance to activate proinflammatory cytokine production and release systemically and locally in the liver [3]. Hepatic oxidative stress and inflammation have been revealed to play critical roles in the progression of NAFLD in recent studies [3, 4]. It is reported that anti-inflammatory therapy can effectively improve the NAFLD/NASH [5]. Besides, gut microbiota was also considered to play an important role in the pathophysiology of NAFLD, through the gut-liver axis [6].

Adenosine monophosphate-activated protein kinase (AMPK) has been proposed to be a potential therapeutic target of NAFLD [7]. As a key energy sensor to alter metabolic pathways, previous studies largely focused on its role on regulation of energy metabolism in related diseases [8, 9]; however, AMPK also took part in the modulation of inflammatory signaling pathways [10]. Recently, attention has shifted toward the role of AMPK on influence of inflammatory degree in metabolic disorders [11], yet its action on alleviating the progression of NAFLD has not been attracted sufficiently. In response to chronic low-grade inflammation induced by high-fat diet (HFD), AMPK activity was found to be reduced in the liver [12]. Moreover, liver-specific AMPK activation would decrease the expression of inflammation genes, which gain improvements in obesity [13]. Besides, it is believed that AMPK exerts a positive influence on Kelch-like ECH-associated protein 1/nuclear factor-related factor 2 (keap1/Nrf2) signaling [14], thus increasing the cellular defense against oxidative and other harmful insults. Accumulating evidence suggests the functional crosstalk between Nrf2 and nuclear factor-*κ*B (NF*κ*B) [15], since the latter is a key transcription factor regulating the cellular response to inflammation. Nevertheless, the related association among AMPK, Nrf2, and NF*κ*B signaling in the liver has not been well investigated in NAFLD. Therefore, we started to examine the crosstalk among AMPK, Nrf2, and NF*κ*B in the alleviation of hepatic oxidative and inflammatory injury in high-fat-induced NAFLD.

Chicoric acid (CA), a major nutraceutical component of chicory (*Cichorium intybus* L.), exhibited a wide range of pharmacological effects including antioxidant, antiviral, anti-inflammatory, and antihyperglycemic activities [16–19]. Although there are few reports revealing the protective effects of chicory seed extract on diabetes- and oleic acid-induced NAFLD [20], information concerning the specific molecular mechanism of CA on HFD-induced NAFLD is rarely available. Growing scientific evidence has demonstrated the regulation of gut microbiota by natural compounds in metabolic disorders which also include NAFLD [21, 22], while the effect of CA on gut microbiota still remains unclear. Overall, the aim of the present study was to investigate the effect and its underlying mechanism of CA on oxidative stress and inflammation in the liver of HFD mice and palmitic acid- (PA-) incubated human hepatoma cell line (HepG2), in addition, to further explore the potential crosstalk among the AMPK, keap1/Nrf2, and NF*κ*B pathways, and to evaluate whether its effects are related to modulations in the gut microbiota of HFD mice.

## 2. Results

### 2.1. CA Mitigated Hyperglycemia, Dyslipidemia, and Systemic Inflammation in Mice Fed with a High-Fat Diet

As illustrated in Figures 1(a) and 1(b), significant higher body weight and white adipose weight were observed in the HFD group in comparison with the ND group (*p* < 0.001). CA (15 and 30 mg/kg) administration significantly reduced body weight and white adipose weight in comparison with the HFD group (*p* < 0.01, *p* < 0.001). Compared with the ND mice, the HFD mice exhibited a significant increase in fasting blood glucose level (*p* < 0.001). Consequently, CA significantly reduced fasting blood level in mice fed with a high-fat diet (Figure 1(c); *p* < 0.001). In addition, compared with the ND mice, serum total cholesterol (TC), triglyceride (TG), and low-density lipoprotein cholesterol (LDL-C) levels were significantly increased, and high-density lipoprotein cholesterol (HDL-C) level was decreased in the HFD mice (*p* < 0.001), while CA administration significantly downregulated TC, TG, and LDL-C levels, as well as upregulated HDL-C level (Figures 1(d)–1(g); *p* < 0.05, *p* < 0.001). Furthermore, the serum levels of interleukin- (IL-) 2, IL-6, IL-1*β*, and tumor necrosis factor- (TNF-) *α* were all increased in the HFD group in comparison with the ND group (*p* < 0.001). Consequently, CA (15 and 30 mg/kg) administration led to the reduction of IL-2 (*p* < 0.01), IL-6 (*p* < 0.001), IL-1*β* (*p* < 0.001), and TNF-*α* (*p* < 0.01, *p* < 0.05). These results suggested that CA could ameliorate HFD-induced hyperglycemia, dyslipidemia, and inflammation in mice.

### 2.2. CA Alleviated Hepatic Lipid Accumulation, Oxidative Stress, and Liver Injury in Mice Fed with a High-Fat Diet

Lipid accumulation in the liver is a sign of NAFLD. As observed in Figure 2(a), Oil Red O- (ORO-) stained lipid droplets were more prominent in sections from the HFD mice in comparison with those of the ND mice, while CA-treated mice had a relative healthier liver tissue (*p* < 0.001). Moreover, large areas of steatosis, cytoplasmic vacuolation (red arrow), and inflammatory cell infiltration (black arrow) were seen in hepatic hematoxylin and eosin (H&E) staining of the HFD mice; all of which were ameliorated after CA treatment (Figure 2(b)). NAFLD activity score analysis also showed the decrease of NAFLD lesion severity by CA (Figure 2(c); *p* < 0.001, *p* < 0.001). The serum MDA level was prominently increased, while the SOD activity was decreased in the HFD group in comparison with those of the ND group (*p* < 0.001), and these parameters were all reversed after CA administration (Figures 2(d) and 2(e); *p* < 0.01, *p* < 0.001). As showed in Figure 2(f), dihydroethidium (DHE) staining of the liver in HFD mice established a distinct higher *in situ* ROS in comparison with the ND mice (*p* < 0.001). However, both two doses of CA treatment notably restored ROS overproduction in the liver (*p* < 0.001). Furthermore, the enzymatic activities of serum pyruvic transaminase/alanine aminotransferase (GPT-ALT) and glutamic oxaloacetic transaminase/aspartate aminotransferase (GOT-AST) were dramatically increased in HFD mice (*p* < 0.001). These two markers of liver injury were both reversed after CA treatment (Figures 2(g) and 2(h); *p* < 0.01, *p* < 0.001). All above data suggested that CA could ameliorate HFD-induced lipid accumulation, oxidative stress, and liver injury.

### 2.3. CA Suppressed the Hepatic NF*κ*B Pathway and Liver Inflammation in HFD Mice

The inflammatory reaction is one of the major features of liver injury in NAFLD [23]. To determine whether CA could inhibit hepatic inflammatory responses in NAFLD, we assessed the hepatic levels of inflammatory cytokines. As showed in Figure 3(a), the hepatic levels of inflammatory cytokines were all increased in the HFD group in comparison with the ND group (*p* < 0.001). Consequently, CA administration reduced IL-2 (*p* < 0.01), IL-6 (*p* < 0.01, *p* < 0.001), IL-1*β* (*p* < 0.01), and TNF-*α* (*p* < 0.05, *p* < 0.05) levels in the liver. As a transcription factor that plays a crucial role in inflammation, NF*κ*B can facilitate the occurrence and development of NAFLD [24]. In parallel with the elevated levels of these inflammatory cytokines, the hepatic protein expression levels of p-IKK*α*/*β* (*p* < 0.01), p-I*κ*B*α* (*p* < 0.01), and p-NF*κ*B (*p* < 0.001) were all significantly increased in HFD mice in comparison with those of ND mice, while CA administration led to a remarkable reduction of these parameters (Figure 3(b); *p* < 0.01). These findings demonstrated the significant anti-inflammatory effect of CA in NAFLD.

### 2.4. CA Ameliorated Lipid Accumulation and Oxidative Stress and Inhibited the NF*κ*B Pathway in PA-Treated HepG2 Cells

To further investigate the role of CA in the amelioration of NAFLD, we constructed an *in vitro* NAFLD model by using HepG2 cells as previously described [25]. As shown in Figure 4(a), there was no significant growth inhibition of HepG2 cells after CA treatment even up to the concentration of 250 *μ*M, indicating the well safety of CA. Significantly more lipid droplets were observed in PA-treated HepG2 cells than those of the normal group (Figure 4(b); *p* < 0.001). And the results showed that the intracellular TC and TG levels were significantly increased in PA-treated HepG2 cells in comparison with the normal group (Figure 4(c); *p* < 0.001). Interestingly, the accumulation of lipids induced by PA treatment was significantly decreased by CA (10 and 20 *μ*M) administration (*p* < 0.01, *p* < 0.001). As showed in Figure 4(d), using DHE and MitoSOX Red staining, we observed that CA reduced the intracellular O_2_^·−^ and mitochondrial oxidative stress in PA-treated HepG2 cells (*p* < 0.001). To further confirm the antioxidant effect of CA in NAFLD, we assessed intracellular ROS through the 2′,7′-dichlorofluorescein diacetate (DCFH-DA) detector. PA treatment significantly elevated ROS production in HepG2 cells, but it was prevented after CA administration (Figure 4(e); *p* < 0.001). In addition, the protein levels of p-IKK*α*/*β* (*p* < 0.01), p-I*κ*B*α* (*p* < 0.001), and p-NF*κ*B (*p* < 0.01) were significantly increased in PA-treated HepG2 cells, which were remarkably decreased after CA administration (Figure 4(f); *p* < 0.01, *p* < 0.001). These data suggested the lipid regulation, antioxidant activity, and the inhibition of the NF*κ*B pathway of CA *in vitro* evaluation.

### 2.5. CA Activated Keap1/Nrf2 Signaling Both in the Liver of HFD Mice and PA-Treated HepG2 Cells

The keap1/Nrf2 pathway is one of the most important defense mechanisms against oxidative stress. It has been shown that Nrf2^−/−^ mice fed with a high-carbohydrate diet failed to induce antioxidant enzymes resulting in oxidative liver damage [26]. In the present study, high keap1 protein level (*p* < 0.01) and low nuclear Nrf2 protein level (*p* < 0.001) were both observed in the liver of HFD mice. In accordance with the inhibition of nuclear Nrf2, significant decreases of protein levels of HO-1 (*p* < 0.001), SOD1 (*p* < 0.01), and SOD2 (*p* < 0.001) were also detected in the liver of HFD mice in comparison with those in ND mice. However, treatment with CA significantly decreased keap1 protein expression level (*p* < 0.05), upregulated nuclear Nrf2 protein level (*p* < 0.001, *p* < 0.01), and increased the protein levels of HO-1 (*p* < 0.01, *p* < 0.001), SOD1 (*p* < 0.001, *p* < 0.01), and SOD2 (*p* < 0.01) in the liver of mice fed with a high-fat diet (Figure 5(a)). In accordance with the suppression of keap1/Nrf2 signaling in the liver of HFD mice, we also observed the elevated keap1 (*p* < 0.05), downregulated nuclear Nrf2 (*p* < 0.001), and decreased HO-1 (*p* < 0.05), SOD1 (*p* < 0.001), and SOD2 (*p* < 0.05) protein levels in PA-treated HepG2 cells, and all of these parameters were reversed to normal after CA administration (Figure 5(b)).

### 2.6. CA Suppressed Oxidative Stress and Inflammation via AMPK Activation

AMPK is a key energy sensor of cellular metabolism, including oxidative stress and inflammation [27, 28]. Both in the liver of HFD mice and PA-treated HepG2 cells, decreased AMPK phosphorylation at threonine 183/172 levels (*p* < 0.01) could be observed in the present study. However, the protein level of p-AMPK was significantly elevated after CA administration both *in vivo* and *in vitro* (Figures 6(a) and 6(b); *p* < 0.05, *p* < 0.01). To further investigate whether CA activates keap1/Nrf2 and inhibits NF*κ*B via AMPK to suppress oxidative stress and inflammation in NAFLD, AMPK activator AICAR and AMPK inhibitor compound C were used as a pair in the CA-mediated action of PA-treated HepG2 cells. The results showed that AICAR (0.5 mmol/L) partly mimicked, while compound C (CC, 10 *μ*mol/L) partly abolished, the downregulative effect of CA on keap1, the upregulative effect of CA on nuclear Nrf2 protein level, and the downregulative effect of CA on NF*κ*B phosphorylation level in PA-treated HepG2 cells (Figures 6(c)). These results suggested that the AMPK pathway was involved in the CA-induced keap1-dependent activation of Nrf2 and suppression of NF*κ*B in PA-treated HepG2 cells.

Moreover, both AICAR and CC were used to investigate whether the AMPK pathway was also involved in the CA-mediated antioxidant effect in PA-treated HepG2 cells. Our data showed that AICAR partly mimicked, while compound C partly abolished the downregulation of CA on ROS production in PA-treated HepG2 cells (Figure 6(d)).

In addition, the Nrf2 inhibitor ML385 (5 *μ*M) partly blocked the upregulation of SOD1, SOD2, and HO-1 and the downregulation of ROS production by CA in PA-induced HepG2 cells. These results indicate Nrf2 as a key factor in the regulation of oxidative stress by CA. Likewise, we investigated whether ML385 blocked the role of CA-mediated NF*κ*B inactivation. The result showed that ML385 diminished CA-induced NF*κ*B suppression, suggesting that Nrf2 plays a key role in CA-mediated amelioration of inflammation (Figures 6(e) and 6(f)).

All these data above demonstrated that CA might suppress oxidative and inflammation via AMPK-mediated keap1/Nrf2 activation and NF*κ*B inhibition in NAFLD.

### 2.7. CA Shaped the Gut Microbiota in HFD Mice

Gut microbiota dysbiosis has been repeatedly observed in NAFLD and NASH [29]. To reveal the possible contribution of gut microbiota in the therapeutic action of CA, we analyzed the fecal microbiota composition using the 16S rRNA pyrosequencing based on V3-V4 region. After size filtering, quality control, and chimera removal, we totally detected 1953854 raw tags from 24 fecal samples with 1953854 clean sequences for further analysis, from which were clustered into operational taxonomic unit (OTU) with similarity higher than 97%. According to the rarefaction curve analysis (Figure 7(a)), the OTU rarefaction curves reached a steady level, indicating that the libraries were large enough to obtain the major information of the bacterial diversity in all samples. A Venn diagram displaying 593 OTUs was shared among 3 groups, and each group owned unique OTUs (Figure 7(b)). Alpha analyses with chao1 (*p* < 0.05), observed_species, PD_whole_tree, and Shannon indexes indicated that the HFD mice had decreased microbial species richness, while CA administration increased the diversity of gut bacteria (Figures 7(c) and 7(d)). The nonmetric multidimensional scaling (NMDS) analysis and principal component analysis (PCA) revealed a separated clustering of gut microbiota among ND, HFD, and CA-treated mice (Figures 7(e) and 7(f)).

The microbial community bar plot analyses on top phylum and genus levels exhibited different bacterial community structures among the groups. The microbial community structure at phylum level was dominated by *Firmicutes* and *Bacteroidetes*. The increased level of the phylum *Firmicutes* and decreased level of the phylum *Bacteroidetes* were observed in HFD mice, which were reversed by CA administration (Figure 8(a)), Thus, *Firmicutes*-to-*Bacteroidetes* ratio (F/B ratio) was significantly increased (*p* < 0.01) in the HFD group compared with the ND group, and after CA administration, this ratio was significantly decreased (Figure 8(b); *p* < 0.05). Among the dominant microbial communities at the genus level, the relative abundance of *Lactobacillus* (*p* < 0.05), *Turicibacter* (*p* < 0.05), *Bacteroides*, *Faecalibaculum* (*p* < 0.001), and *Candidatus_Saccharimonas* was higher, while the proportion of *Lachnospiraceae*, *Allobaculum*, *Ruminococcaceae_UCG-014*, and *Alloprevotella* was decreased in HFD mice compared with the ND mice. However, CA administration reversed the proportion of *Lactobacillus* (*p* < 0.05), *Turicibacter* (*p* < 0.05), *Ruminococcaceae_UCG-014*, *Alloprevotella*, and *Candidatus_Saccharimonas* in HFD mice (Figure 8(c)). The community heat map analysis confirmed these changes (Figure 8(d)). All these suggested that CA enhanced the diversity of gut microbiota and restored the alert microbiota to a state more similar to ND mice.

## 3. Discussion

Oxidative stress, inflammatory response, and gut microbiota are critical factors in the progression of NAFLD. Due to its potential antioxidant and anti-inflammatory activities, CA may contribute to the intervention of NAFLD. In the present study, we evaluated the effects of CA treatment on NAFLD both in HFD mice and PA-induced HepG2 cells. The amelioration of oxidative stress and inflammation was observed. Moreover, CA greatly shaped the composition of gut microbiota into a status more similar to ND mice. Collectively, the therapeutic effect of CA on NAFLD has been proven through the present investigation.

As an important cellular sensor to restore cellular energy homeostasis and a central regulator of multiple metabolic pathways, AMPK has been proposed as a therapeutic target for metabolic diseases [7, 30, 31]. The ability to control the energy balance equation through defined metabolic pathways heavily pursues AMPK as a golden target against obesity [31]. Activation of AMPK by the E3 ubiquitin ligase makorin ring finger protein 1 (MKRN1) represses diet-induced metabolic syndrome [8]. Lipid metabolism abnormal and insulin resistance are two typical features of NAFLD, so the regulative effects of lipid and glucose metabolism of AMPK have got the most attention in NAFLD. Liver-specific reduction of AMPK activity inhibits acetyl-CoA carboxylase (ACC) phosphorylation and leads to lipogenesis increases in hepatocytes [9]. Liver AMPK activator PF-06409577 decreases both hepatic and systemic lipids in the high-fat-diet-induced NAFLD models of the rodent and monkey preclinical models [32]. Activation of AMPK suppresses hepatic glucose release and enhances insulin sensitivity in dexamethasone-induced fatty liver disease in C57BL/6 mice [33]. In this study, the reduction of AMPK phosphorylation was observed both in the liver of HFD mice and PA-treated HepG2 cells, in company with elevated body weight, serum glucose, and lipid metabolism disorders. It has been surmised that numerous polyphenols are capable of activating AMPK via the elevation of AMP levels by inhibiting mitochondrial ATP production, which serves as indirect AMPK activators [34]. CA has been found to restore insulin signaling and dyslipidemia [19, 35]. Our results indicated that CA alleviated HFD-induced hyperglycemia and dyslipidemia in mice, as well as reduced lipid accumulation in the liver. In addition to these, CA could also restore PA-induced lipid drop deposition and decrease TC and TG levels in HepG2 cells. Importantly, decreased AMPK phosphorylation levels in the liver of HFD mice and PA-treated HepG2 cells were both reversed by CA.

Moreover, oxidative metabolism also contributes to oxidative stress and inflammation during NAFLD [36]. Recent researches demonstrated that suppression of oxidative stress and inflammation contributed to the amelioration of NAFLD or NASH [5, 37, 38]. Not only as a key sensor of energy balance but also a factor of redox balance improvement and inflammation reduction, the antioxidation and anti-inflammatory effect of AMPK activation has gained more attention [39, 40]. Activation of AMPK could alleviate mitochondrial oxidative damage and apoptosis [40]. AMPK was also reported to prevent oxidative stress-induced senescence by improving autophagic flux and NAD(+) homeostasis [41]. Furthermore, stimulation of AMPK phosphorylation prevented HFD-induced insulin resistance and inflammation in adipose tissue through anti-inflammatory effects in obesity and attenuated lipopolysaccharide-induced secretion of proinflammatory cytokines such as TNF-*α* and MCP-1 [11]. In this study, we observed oxidative stress and inflammation, including elevated MDA and suppressed SOD activity in HFD mice, overproduction of O_2_^·−^ in the liver and ROS in PA-treated HepG2 cells, and increased serum IL-2, IL-6, IL-1*β*, and TNF-*α* levels in HFD mice. It has been noted that the antioxidant and anti-inflammatory effects of CA have already been documented in metabolic diseases, including obesity and atherosclerosis [16, 42]. Consistent with these reports, in our experiments, CA treatment dramatically decreased ROS production and inflammatory cytokines. Taken together, our data demonstrated that CA could mitigate high-fat-induced inflammation and oxidative damage *in vivo* and *in vitro* probably via AMPK phosphorylation activation.

Importantly, those benefits of antioxidative and anti-inflammation were also observed in previous studies on Nrf2 activation [43–45]. Keap1/Nrf2 system forms the cellular defense against oxidative and electrophilic stresses, which has been known to attenuate inflammation [44, 45]. Activation of Nrf2 has also been confirmed to reduce hepatic lipid accumulation in bisphenol A-induced mouse model of NAFLD [46]. It has been demonstrated that Nrf2-dependent antioxidant genes contain almost all the antioxidant enzymes, including SOD, catalase, glutathione S-transferase (GST), glutathione peroxidase-1 (GPX-1), and HO-1 [47]. Activation of Nrf2 in hepatocytes inhibited inflammatory and oxidative stress, suppressed hepatic steatosis, and mitigated liver fibrosis in NASH [48, 49], while inactivation of Nrf2 led to aggravation of liver injury in NASH; thus, impairment of Nrf2 activity represented a major risk factor for the evolution of NAFLD to NASH [50]. We surmised that activation of Nrf2 functions attributed to ROS elimination in NAFLD. Likewise, we observed keap1 and Nrf2 alteration both in the liver of HFD mice and PA-treated HepG2 cells. Activation of Nrf2 by CA increased the expression of downstream antioxidant genes, including SOD1, SOD2, and HO-1, thereby functionally attenuated hepatocyte injury *in vivo* and *in vitro*. What is interesting, recent researches have revealed the crosstalk between AMPK and Nrf2 [14, 39, 51]. Nrf2 signaling was revealed as the downstream signal of AMPK in oxidative stress and inflammation [39], and AMPK activation promotes autophagic degradation of keap1 to induce Nrf2 dissociate from keap1 and translocate to the nucleus [52]. However, whether Nrf2 is the downstream signal of AMPK in HFD-induced NAFLD still remains unclear. To confirm the crosstalk between AMPK and Nrf2 in NAFLD and whether CA could regulate Nrf2 via AMPK, we conducted AMPK activator AICAR and inhibitor compound C in PA-induced HepG2 cell. Our results showed that both PA-induced elevation of keap1 and reduction of nuclear Nrf2 protein level and ROS overproduction in HepG2 cells were reversed by either CA or partly reversed by AMPK activator AICAR. Importantly, the downregulative effect on keap1 level and upregulative effect on Nrf2 level of CA and the decease of ROS production were partly eliminated by adding AMPK inhibitor compound C. These results indicated that the AMPK pathway was involved in the keap1-depedent regulation of CA on Nrf2 level in PA-treated HepG2 cells. Likewise, the upregulative effect on SOD1, SOD2, and p-NF*κ*B protein levels, and the downregualtive effect of ROS production of CA were party diminished by Nrf2 inhibitor ML385. These results further indicated that Nrf2 was involved in CA-mediated amelioration of oxidative stress in PA-treated HepG2 cells.

On the one hand, inflammation results in a stress response of hepatocytes and may lead to lipid accumulation and precede steatosis [53]. On the other hand, increased FFA levels, insulin resistance, and adipose tissue dysfunction activate the production and release of proinflammatory cytokines, both systemically and locally in the liver [3]. NF*κ*B has been recognized as a key proinflammatory transcription faction in inflammation and immune response. Persistent NF*κ*B pathway activation has been shown in animal models or patients with NAFLD and NASH [54–57]. To further characterize the mechanism of inhibitory effect of CA on inflammatory cytokine production, we investigated the effect of CA on the NF*κ*B pathways and serum inflammatory cytokines in HFD mice. It was well noted that the increase of serum IL-2, IL-6, IL-1*β*, and TNF-*α* was confirmed in HFD mice, as well as the inflammatory cell infiltration detected by liver H&E staining. CA treatment significantly downregulated inflammation systemically and in the liver. Studies have shown that the NF*κ*B pathway could be regulated by AMPK and Nrf2 [15, 58]. Herewith, we showed many degrees of upregulation on NF*κ*B phosphorylation by AICAR in PA-treated HepG2 cells. Moreover, the upregulative effect of CA on NF*κ*B phosphorylation level was partly eliminated by compound C. Similarly, the suppression on p-NF*κ*B of CA was party diminished by ML385. These results indicated that the AMPK-Nrf2 pathway was involved in the regulation of CA on NF*κ*B suppression in PA-treated HepG2 cells.

Growing evidences indicate the gut microbiota alteration in metabolic disorders, including NAFLD [29]. In the present study, the composition and proportion of gut microbiota were changed in HFD mice. Our 16S rRNA sequencing experiment revealed that CA treatment increased the OTU numbers and upregulated chao1, observed_species, PD_whole_tree, and Shannon indexes in HFD mice. Based on the NMDS and PCoA, HFD changed the overall gut microbiota composition in NAFLD mice, and it was reversed by CA treatment. *Bacteroidetes* and *Firmicutes* are two dominant bacterial divisions in the gut, and numerous studies have observed that the ratio of *Firmicutes* to *Bacteroidetes* in gut microbiota, characteristic of “obese microbiota”, was associated with metabolic disorders including obesity and NAFLD [22, 59, 60]. In the current study, HFD induced relative increase of *Firmicutes* and decrease of *Bacteroidetes* in the gut in comparison with the ND mouse group, causing the significantly elevation of F/B ratio, in parallel with body weight gain and adiposity in HFD mice. CA treatment significantly reversed F/B ratio in HFD mice, as well as decreased HFD-induced body weight gain and adiposity. Although *Lactobacillus* is recognized as a probiotic bacterium in metabolic disorders including NAFLD, some studies showed the contrary results [61–63]. Elevated *Lactobacillus* in the gut may correlate with decreased insulin sensitivity and increased plasma inflammatory cytokine [61]. Similar increase of *Lactobacillus* was also observed in NAFLD patient and mice [62, 63]. Furthermore, some species of *Lactobacillus* such as *L. reuteri* also had a redundant role associated with increased body fat and insulin levels [64]. In the current study, the proportion of *Lactobacillus* was increased almost 3 folds (from 5.3% to 14%) in HFD mice in comparison of ND mice and lowered to 6.1% after CA administration. NAFLD severity associates with gut dysbiosis and a shift in metabolic function of the gut microbiota. We conjectured that overmuch or disproportionate *Lactobacillus* might cause adverse reactions. *Bacteroides* abundance was significantly increased in NASH and has been defined as independently associated with NASH [65]. In this study, *Bacteroides* was increased in the HFD group, indicating the high severity of NAFLD in the mice. *Turicibacter*, a genus of the *Firmicutes* phylum *Firmicutes*, has been primary confirmed to alter gut microbiota of healthy and be associated with hyperlipidemia and body gain [66]. Compared with the HFD group, the abundance of *Turicibacter* was decreased in the CA group. *Faecalibaculum* belonging to *Erysipelotrichaceae*, enriched in HFD mice, was closely related to adiposity and found as biomarker correlated with oxidative stress [67]. In this study, the amount of *Faecalibaculum* was increased in HFD mice and reversed to normal after CA administration. CA also contributed to an increase in the abundance of *Alloprevotella*, which was associated with health benefits in short-chain fatty acids producing and anti-inflammatory [68]. We primary infer that the amelioration of NAFLD by CA may be associated with the alleviation on the dysbiosis of gut microbial, and further investigation is needed to support this hypothesis.

We noticed that previous studies also tried to explore the therapeutic effect of CA on NAFLD or NASH, and many researches had been well done. Using methionine and choline deficiency-induced mouse model and cell models, Kim et al. revealed the improvement of NASH by CA [69]. Xiao et al. placed emphasis on the antiobesity effect of CA by the regulation of COX-2, p-JNK, PPAR*γ*, and C/EBP*α* in high-fat-diet mice [70]. Here, using high-fat-diet-induced NAFLD mouse model and PA-induced cell model, we focused on the antioxidant and anti-inflammation effect of CA and tried to connect and explain the crosstalk among AMPK, keap1/Nrf2, and NF*κ*B system in HFD-induced NAFLD for the first time. These results of the study formed a completed signal path loop, which clearly figured out the mechanism of CA on HFD-induced NAFLD. Additionally, we applied high-throughput pyrosequencing of 16S rRNA to observe the changes of related gut microbial composition, and the results suggested that high-fat-diet-induced decrease of *Firmicutes*-to-*Bacteroidetes* ratio and dysbiosis of NAFLD mice could be reversed by CA treatment. Ziamajidi et al. observed that chicory seed extract improved diabetes- and oleic acid-induced NAFLD and NASH by PPAR*α* and SREBP-1 [20]. Chicory seed extract contains a variety of compounds, yet the precise ingredient is not clear. Here, in this study, we confirmed the amelioration of NAFLD by CA, as a single active compound. Mohammadi et al. paid the attention on the improvement of lipid accumulation by CA and fish oil through a NAFLD cell model via the AMPK-mediated SREBP-1/FAS and PPAR*α*/UCP2 pathways [71]. Here, we investigated the improvement of oxidative stress and inflammation in both NAFLD animal and cell models via the AMPK/Nrf2/NF*κ*B pathway and this might be associated with the restored gut microbiota. The pathogenesis of NAFLD is very complex, and CA may serve as a multitargeting pharmacologically active compound. Combined with these previous studies, CA would be an attractive agent for the amelioration of NAFLD.

In conclusion, CA treatment displays an effect against lipid dysregulation, oxidative stress, inflammation, and gut microbiota in NAFLD. The action of CA in upregulating AMPK phosphorylation and nuclear Nrf2 level, as well as suppression of NF*κ*B in hepatocytes, may contribute to the protective effect of the liver in NAFLD. It is conceivable that CA may be able to protect hepatocytes from oxidative damage and inflammation via regulating AMPK-mediated Nrf2 activation and NF*κ*B inactivation and shaping gut microbiota. Our findings provide strong scientific basis of CA for amelioration of NAFLD and its related metabolic diseases.

## 4. Materials and Methods

### 4.1. Reagents and Chemical

CA (purity > 98%), palmitic acid, and fatty acid-free bovine serum albumin (BSA) were purchased from Nanjing Spring & Autumn Biological Engineering Corporation (Nanjing, China), Macklin (Shanghai, China), and YEASEN (Shanghai, China), respectively. AIACAR, Compound C, and ML385 were obtained from Beyotime Institute of Biotechnology (Haimen, China), Selleck (Houston, TX, USA), and MedChemExpress (NJ, USA), respectively. Dulbecco's modified Eagle's medium (DMEM), penicillin-streptomycin, and fetal bovine serum (FBS) were all obtained from Invitrogen-Gibco (Grand Island, NY). Cell Counting Kit-8 (CCK-8) assay and bicinchoninic acid (BCA) Protein Quantification Kit were purchased from Biosharp (Hefei, China). Biochemical indexes including glucose, TC, TG, LDL-C, HDL-C, GPT-ALT, and GOT-AST assay kits were purchased from Nanjing Jiancheng Bioengineering Institute (Jiangsu, China). MDA and SOD assay kits, DHE and DCFH-DA probes, and the nuclear protein extraction kit were offered by Beyotime Institute of Biotechnology (Jiangsu, China). ORO staining kit was purchased from Nanjing Jiancheng Bioengineering Institute (Jiangsu, China). MitoSOX Red probe was obtained from Yeasen (Shanghai, China). Serum and hepatic inflammatory cytokines including IL-2 (EK202HS-96), IL-6 (EK206/3-96), IL-1*β* (EK201B/3-96), and TNF-*α* (EK282HS-96) enzyme-linked immunosorbent assay (ELISA) kits were purchased from MultiSciences (Lianke) Biotech Co., Ltd (Zhejiang, China). Antibodies against Nrf2, NF*κ*B, p-NF*κ*B, I*κ*B*α*, p-I*κ*B*α*, IKK*β*, p-IKK*α*/*β*, and the HRP-linked secondary antibodies were obtained from Cell Signaling (Boston, MA, USA); antibodies against keap1, SOD1, and HO-1 were obtained from Santa Cruz Biotechnology (CA, USA); antibodies against SOD2 and AMPK were purchased from Proteintech Group (Chicago, USA). p-AMPK (T183/172) was purchased from Bioworld Technology (MN, USA).

### 4.2. Animal Model and the Treatment

All animal experiments were in strict accordance with the *Guide for the Care and Use of Laboratory Animals* approved by the Animal Ethics Committee of China Pharmaceutical University (certificate number: SYXK2016-0011, approval date: 27 January 2016 to 26 January 2021). Male C57BL/6 mice (20 to 25 g body weight) were housed with food and water available *ad libitum* in light, temperature, and humidity-controlled environments. The normal control group was fed with normal diet (ND), while the others were fed with HFD (18% lard stearin (*w*/*w*), 5% egg powder, 1% cholesterol, 20% sucrose, 0.1% bile salt, and 55.9% normal diet) [72] for 9 weeks. Then, the HFD mice received either CA (15 or 30 mg/kg/d, dissolved in water) or saline solution daily for 9 weeks by gavage (*n* = 8). Mice were sacrificed, and then the blood samples were collected from the carotid artery and centrifuged to obtain serum, and the livers were harvested for the following biochemical analysis. The serum and liver tissues were stored at -80°C.

### 4.3. Detection of Serum Biomarkers

The levels of serum glucose, TC, TG, LDL-C, HDL-C, MDA, SOD activity, GPT-ALT, and GOT-AST were determined by commercial assay kits in accordance with the manufacturer's instructions. The inflammatory cytokines including IL-2, IL-6, IL-1*β*, and TNF-*α* were measured using ELISA kits in accordance with the manufacturer's instructions.

### 4.4. Histological Assessment

Pieces of the liver were fixed in 4% paraformaldehyde and processed to paraffin wax then stained with hematoxylin and eosin (H&E). In addition, lipid droplets in the liver were observed by ORO staining in the frozen liver sections and quantified by ImageJ software. Histopathological changes of the livers were observed and photographed under a light microscope (Olympus, Tokyo, Japan).

### 4.5. Measurement of Hepatic Inflammatory Cytokines

Liver tissues were homogenized in lysis buffer (pH 7.2, Tris with 1% Triton X-100 and 0.1% protease inhibitor) and centrifuged at 12,000 *g* for 15 min. The supernatants were collected for determination of IL-2, IL-6, IL-1*β*, and TNF-*α* by ELISA kits according to the manufacturer's instructions adjusted for protein content.

### 4.6. Cell Culture and Treatment

HepG2 cells were obtained from FuHeng Cell Center, Shanghai, China. Cells were cultured in low-glucose DMEM supplemented with 5% FBS and 1% penicillin-streptomycin and incubated at 37°C and 5% CO_2_. PA was dissolved in 50% ethanol by heating at 50°C, then conjugated with 10.5% fatty acid-free BSA (volume ratio 1 : 25) under agitation at 40°C for 2 h, and finally diluted in culture media. HepG2 cells were pretreated with or without 250 *μ*M PA for 24 h and then incubated in the culture media with or without 250 *μ*M PA or CA (10 and 20 *μ*M, dissolved in PBS) for another 24 h. To clarify the involved signaling pathways, AICAR (0.5 mM) or compound C (10 *μ*M) was used to treat HepG2 cells.

### 4.7. Cell Viability Analysis

The cell viabilities were assessed using CCK-8 assay. In brief, HepG2 cells were plated into 96-well plates with 2 × 10^5^ per well and incubated overnight. Afterwards, the cells were incubated with different concentrations (0-250 *μ*M) of CA for 24 h. Subsequently, CCK-8 working solution was added to each well and cultivated for another 1 h. The absorbance was recorded on a microplate reader at 450 nm (Molecular Devices, Sunnyvale, USA).

### 4.8. Measurement of Lipid Uptake in HepG2 Cells

The cells were homogenized in lysis buffer. The intracellular TC and TG contents were measured using commercially assay kits according to the manufacturer's instructions. The protein concentration was assayed using BCA protein quantitative kit. The intracellular TC and TG contents were presented as *μ*mol/mg protein.

The lipid deposition in HepG2 cells was measured by ORO staining [73]. Briefly, after fixed in 4% formaldehyde for 15 min fixation and then cleaned with PBS, ORO working solution was injected into cells for 30 min. The cells were immediately washed with 60% isopropanol, incubated with hematoxylin for 5 minutes, washed by PBS and immediately imaged using microscopy (Olympus, Tokyo, Japan), and quantified by ImageJ software.

### 4.9. Detection of ROS

Liver in situ O_2_^·−^ production was determined by fluorescence probe DHE labeling. Frozen liver sections were prepared for immediate DHE staining. Thawed sections were incubated with 2 *μ*M DHE at 37°C for 30 minutes (avoiding light). After washed 3 times by PBS, sections were immediately imaged using fluorescence microscopy (Olympus, Tokyo, Japan) and quantified by ImageJ software.

Intracellular O_2_^·−^ levels were detected using the DHE staining. Cells were incubated with PBS diluted DHE (10 *μ*M) at 37°C for 20 min (avoiding light), washed with PBS for 3 times, and then imaged using fluorescence microscopy (Olympus, Tokyo, Japan). Mitochondrial ROS in HepG2 cells was measured by MitoSOX Red at a concentration of 4 *μ*M for 20 min at 37°C, imaged using fluorescence microscopy (Olympus, Tokyo, Japan), and quantified by ImageJ software.

DCFH-DA fluorescent probe was used to detect intracellular ROS generation. Cells were washed with PBS after incubation with DCFH-DA (10 *μ*M) at 37°C for 30 min (avoiding light). Fluorescence intensity was measured at 530 nm with an excitation wavelength of 485 nm using a fluorescence microscope (Tecan, Crailsheim, Germany).

### 4.10. Western Blot

The liver tissues and HepG2 cell cultures were lysed in RIPA buffer and then centrifuged again at 12,000 *g* for 15 min at 4°C, following the supernatant collection. The nuclear protein was obtained using a nuclear protein extraction kit. The concentration of protein was measured using a BCA protein assay kit, and then the protein level was normalized and the 5× loading buffer was added, following boiled at 100°C.

The proteins (equal amount) were electrophoresed on 10% SDS-PAGE at 85 V (stacking gel) and 135 V (separating gel), transferred onto a 2.2 *μ*M PVDF membrane in a 4°C refrigerator at 300 mA for 1.5 h, blocked with 5% skim milk for 2 h at room temperature, and incubated with primary antibodies overnight at 4°C. The membranes were washed three times with TBST (8 min each time) and then probed with horseradish peroxidase- (HRP-) conjugated anti-rabbit or anti-mouse secondary antibody for 1 h followed by six washes with TBST (8 min each time). The blot bands were visualized using enhanced chemiluminescence, and band intensities were analyzed using ImageJ gel analysis software. *β*-Actin and histone H3 were used as the loading controls.

### 4.11. Gut Microbiota Analysis

At the end of the intervention period, fresh fecal samples were collected and stored at -80°C immediately. The DNA of fecal samples was extracted using an EZNA Stool DNA kit (Omega Bio-tek, Norcross, GA, USA) according to the manufacturer's instructions. Purity and quality of the genomic DNA were checked on 0.8% agarose gels. Amplification was performed targeting the variable regions V3-4 of bacterial 16S rRNA gene with the primers 338F (ACTCCTACGGGAGGCAGCAG) and 806R (GGACTACHVGGGTWTCTAAT). The PCR was carried out on a Mastercycler Gradient (Eppendorf, Germany) in triplicate: 25 *μ*L mixture containing 12.5 *μ*L of KAPA 2G Robust Hot Start Ready Mix, 1 *μ*L of forward primer (5 *μ*M), 1 *μ*L of reverse primer (5 *μ*M), 5 *μ*L of DNA sample (30 ng), and 5.5 *μ*L of H_2_O. Cycling parameters were 95°C for 5 min, followed by 28 cycles of 95°C for 45 s, 55°C for 50 s, and 72°C for 45 s with a final extension at 72°C for 10 min. The PCR products were purified using a QIAquick Gel Extraction Kit (QIAGEN, Germany) and quantified using real-time PCR. Deep sequencing was performed at Beijing Allwegene Technology Inc. (Beijing, China) using Illumina Miseq PE300 sequencing platform (Illumina, San Diego, CA, USA) as described previously [74].

### 4.12. Statistical Analysis

All statistical analyses were performed using GraphPad Prism 8 (San Diego, CA). All data were expressed as the mean ± standard error of the mean (SEM). Statistical analysis was performed by one-way ANOVA analysis followed by Dunnett's post hoc test. Statistical significance was set at *p* < 0.05.

## Figures and Tables

**Figure 1:** Effects of CA on hyperglycemia, dyslipidemia, and inflammation in HFD mice. CA affected body weight (a), white adipose (b), blood glucose (c), serum TC (d), TG (e), HDL-C (f), LDL-C (g), and serum inflammatory cytokines (h) in HFD-fed mice. C57BL/6 mice were randomly divided into four groups: in the ND group, mice were fed with a ND and received 0.9% NaCl solution. In the HFD group, mice were fed with a HFD diet and received 0.9% NaCl solution. In the two HFD+CA groups, mice were fed with a HFD and received 15 mg/kg or 30 mg/kg of CA once daily by oral gavage. Data represent the mean ± SEM, *n* = 8 per group. ^+++^*p* < 0.001 vs. ND group. ^∗^*p* < 0.05, ^∗∗^*p* < 0.01, and ^∗∗∗^*p* < 0.001 vs. HFD group.

**Figure 2:** CA alleviated hepatic lipid accumulation, oxidative stress, inflammation, and liver injury in HFD-fed mice. (a) Hepatic ORO staining (scale bar: 100 *μ*M) and quantitative analysis of lipid content (*n* = 6). (b) Histological analysis of liver tissues by H&E staining (scale bar: 100 *μ*M); red arrow: cytoplasmic vacuolation; black arrow: inflammatory cell infiltration. (c) NAFLD activity score determined according to the liver section histology analysis (*n* = 6). (d, e) Serum SOD and MDA activity levels in mice (*n* = 8). (f) The *in situ* ROS of the liver detected by DHE staining (scale bar: 50 *μ*M) and the fluorescence intensity analysis (*n* = 4). (g, h) Serum GPT-ALT and GOT-AST levels in mice (*n* = 8). Data represent the mean ± SEM. ^++^*p* < 0.01 and ^+++^*p* < 0.001 vs. ND group. ^∗∗^*p* < 0.01 and ^∗∗∗^*p* < 0.001 vs. HFD group.

**Figure 3:** CA suppressed the hepatic NF*κ*B pathway and liver inflammation in HFD mice. (a) Hepatic levels of IL-2, IL-6, IL-1*β*, and TNF-*α* (*n* = 8). (b) Hepatic p-IKK*α*/*β*, p-I*κ*B*α*, and p-NF*κ*B protein levels in mice (*n* = 3). Data represent the mean ± SEM. ^++^*p* < 0.01 and ^+++^*p* < 0.001 vs. ND group. ^∗^*p* < 0.05, ^∗∗^*p* < 0.01, and ^∗∗∗^*p* < 0.001 vs. HFD group.

**Figure 4:** CA ameliorated lipid accumulation and oxidative stress, as well as inhibited the NF*κ*B pathway in PA-induced HepG2 cells. (a) Cell viability after treatment with different concentrations of CA from 0 to 250 *μ*M for 24 h (*n* = 8). (b) lipid droplets detected by ORO staining (scale bar: 100 *μ*M) and quantitative analysis of lipid content in HepG2 cells (*n* = 4). (c) Intracellular TC and TG levels in HepG2 cells (*n* = 8). (d) The intracellular O_2_^·−^ and mitochondrial ROS detected by DHE (scale bar: 100 *μ*M), MitoSOX Red staining (scale bar: 50 *μ*M), and the fluorescence intensity analyses in PA-treated HepG2 cells (*n* = 8). (e) ROS production detected by DCFH-DA detector (*n* = 8). (f) The protein levels of p-IKK*α*/*β*, p-I*κ*B*α*, and p-NF*κ*B in HepG2 cells (*n* = 3). Data represent the mean ± SEM. ^++^*p* < 0.01 and ^+++^*p* < 0.001 vs. normal group. ^∗∗^*p* < 0.01 and ^∗∗∗^*p* < 0.001 vs. PA group.

**Figure 5:** CA regulated keap1/Nrf2 signaling in the liver of HFD mice and PA-treated HepG2 cells. (a, b) The protein levels of keap1, nuclear Nrf2, SOD1, SOD2, and HO-1 in the liver or HepG2 cells. Data represent the mean ± SEM, *n* = 3 per group. ^++^*p* < 0.01 and ^+++^*p* < 0.001 vs. ND or normal group. ^∗∗^*p* < 0.01 and ^∗∗∗^*p* < 0.001 vs. HFD or PA group.

**Figure 6:** CA suppressed oxidative stress and inflammation via AMPK activation. (a, b) Effects of CA on the phosphorylation of APMK in the liver and HepG2 cells (*n* = 3). (c) The protein levels of keap1, nuclear Nrf2, and p-NF*κ*B in HepG2 cells (*n* = 3). (d) ROS production of cells detected by DHE staining (scale bar: 100 *μ*M) and the fluorescence intensity analysis (*n* = 4). (e) The protein levels of SOD1, SOD2, HO-1, and p-NF*κ*B in HepG2 cells (*n* = 3). (f) ROS production in HepG2 cells detected by DCFH-DA detector (*n* = 8). Data represent the mean ± SEM. ^++^*p* < 0.01 and ^+++^*p* < 0.001 vs. ND or normal group. ^∗^*p* < 0.05 and ^∗∗^*p* < 0.01 vs. HFD or PA group.

**Figure 7:** Effect of CA (30 mg/kg) treatment on the relative abundance of gut microbial community in HFD mice. (a) Rarefaction curve for each sample (ND1-ND8: mice fed with a ND and received 0.9% NaCl solution; HFD1-8: mice fed with a HFD diet and received 0.9% NaCl solution; CA1-8: mice fed with a HFD and received 30 mg/kg of CA once daily by oral gavage). (b) Venn diagram of the overlap of the OTUs in the gut microbiota in different treatments. (c) The bacterial richness in gut estimated by alpha-diversity of chao1, observed_species, PD_whole_tree, and Shannon indexes. The *β*-diversity analysis of nonmetric multidimensional scaling (NMDS) (d) and principle coordinate analysis (PCoA) (e). Data represent the mean ± SEM, *n* = 8. ^+^*p* < 0.05 vs. ND group.

**Figure 8:** Effect of CA treatment on the population structure of gut microbiota in HFD mice. (a) Bar plot analysis of microbial community at the phylum level in mice. (b) The alteration in the Firmicutes-to-Bacteroidetes ratio in mice. Bar plot analysis (c) and heat map analysis (d) of microbial community at the genus level in mice. Data represent the mean ± SEM, *n* = 8 per group. ^++^*p* < 0.001 vs. ND group. ^∗^*p* < 0.05 vs. HFD group.

## Data Availability

The data used to support the findings of this study are available from the corresponding author upon request.
